# Role of Bioinformatics Analysis in Early Differential Diagnosis of Ovarian Cancer

This article has been retracted.

**DOI:** 10.1155/2022/6129817

**Published:** 2022-09-16

**Authors:** Lihua Zhang, Yuanyuan Zhao, Li Li, Huadong Xin

**Affiliations:** The Second Department of Gynaecology, Central Hospital of City Handan, Handan 056001, Hebei, China

## Abstract

In order to solve the problem of early differential diagnosis of ovarian cancer, this paper proposes the role of bioinformatics analysis in early differential diagnosis of ovarian cancer. This method uses bioinformatics methods to mine the existing data in the tumor database and obtain tumor-related molecules. It is an efficient method to obtain effective biomarkers, screen signal pathway molecules, and reveal the internal mechanism of tumor occurrence and development. Using this method can greatly improve the efficiency and reliability of screening diagnosis, prognosis, and treatment targets. The results showed that 5821 new lncRNA transcripts and 4611 new lncRNA genes were identified by lncScore from the assembled transcripts. 10 new lncRNA transcripts and 174 new lncRNA genes were found to be differentially expressed in ovarian cancer.

## 1. Introduction

Currently, the standard treatment for ovarian cancer is cytoreductive surgery and adjuvant therapy. Chemotherapy drugs for ovarian cancer mainly include platinum chemotherapy drugs including cisplatin, carboplatin, and oxaliplatin and poly(ADP-ribose) polymerase (PARP) inhibitors including olaparib, niraparib, veliparib, and rucaparib. Although PARP inhibitors have achieved certain efficacy in the treatment of ovarian cancer, and new targeted therapies for ovarian cancer are constantly being developed, due to the problems of low response rate and drug resistance, a considerable number of patients are still difficult to benefit from the existing targeted therapies, and the high mortality rate of ovarian cancer has not been fundamentally changed.

## 2. Literature Review

Ovarian cancer is one of the most common malignancies of the female reproductive system, according to Medhat et al. Because its early symptoms are not obvious, nearly 60% of ovarian cancer is in the advanced stage when it is diagnosed, and the mortality is very high [1].Therefore, early detection of ovarian cancer is the key to effective treatment. In addition, LBCR and others found that the prognosis of ovarian cancer (especially ovarian serous cystadenocarcinoma) is very poor due to the high recurrence and metastasis rate of ovarian cancer after surgery and chemotherapy resistance, and the residence is the first gynecological malignant tumor [2]. Jiang et al. found that, in order to study the early diagnosis and clinical treatment of ovarian cancer, it is necessary to understand its occurrence and development and the molecular mechanism of drug resistance [3]. At present, Li et al. found that using high-throughput sequencing technology, a large number of long-chain noncoding RNAs (lncRNAs) with maladjusted expression in ovarian cancer have been found, but the function and mechanism of most lncRNAs in ovarian cancer are still unclear [4]. lncRNA has high tissue and space-time expression specificity and diverse functions and has become a research hotspot in the field of ovarian cancer. Wang et al. were able to identify ovarian cancer-related lncRNAs through systems biology and bioinformatics methods, build an lncRNA regulatory network, and deeply explore the function of lncRNA and its molecular mechanism in ovarian cancer with the accumulation of ovarian cancer transcriptome data and the implementation of cancer gene mapping (TCGA) program in recent years [5]. Wu et al. found that the current transcript assembly based on high-throughput sequencing data still has problems such as poor assembly quality and loss of start or stop codons, which makes incomplete encoded transcripts easy to be misclassified as lncRNA [6]. Therefore, they proposed a new lncRNA recognition tool lncScore. This tool was superior to other tools (such as CPAT and CNCI) in accurately distinguishing between lncRNA and mRNA. Especially in the classification of incomplete coding transcripts, the recognition accuracy is more than 95%. lncScore also has the advantages of supporting multithreading, short time, and high efficiency. In addition, Chenget al. extracted ovarian cancer and adjacent tissues and sequenced the transcriptome. From the assembled transcripts, 5821 new lncRNA transcripts and 4611 new lncRNA genes were identified by lncScore, of which 10 new lncRNA transcripts and 174 new lncRNA genes were found to be differentially expressed in ovarian cancer [7]. Liang et al. found the existing methods based on the overall expression correlation to screen lncRNA-miRNA-mRNA competitive triples are greatly affected by the sample set and can only screen miRNA central candidate triples [8]. A new competitive triplet recognition tool, LncMiM, is proposed. Using the improved sliding window method, the tool can screen three central candidate triples based on the change of expression correlation at the local level, which not only reduces the false-positive rate of competitive triples but also improves the sensitivity of recognition. Gisonno et al. found that based on the high-throughput sequencing data of 373 patients with ovarian cancer in TCGA database, an lncRNA regulatory network was constructed using the competitive triples identified by LncMiM, and its function was analyzed [9]. The results showed that the regulatory network was closely related to the proliferation, division, and migration of ovarian cancer cells. Deng et al. found that the internal ribosomal entry site (IRES) functional element contained in RNA usually mediates the cap-independent RNA translation mechanism. Recently, it has been found that it plays an important role in the formation and development of cancer. A complete IRES functional element database is urgently needed [10]. Therefore, we manually collected all the experimentally verified IRES components from the literature and constructed a new IRES database IRESbase. There are 1184 IRES entries in this database, eight times more than other databases, and the annotation information is more abundant, especially the genome location information of human IRES elements. Based on the high-throughput sequencing data of ovarian cancer in TCGA database, we analyzed the interaction between lncRNA and mRNA containing the IRES element, screened 110 lncRNAs related to the expression of mRNA containing the IRES element, and predicted their potential functions. The results suggest that these lncRNAs may affect the proliferation of ovarian cancer cells by regulating the cell cycle and metabolic process and affect the migration of ovarian cancer cells by regulating the Slit/Robo signal pathway. The role of bioinformatics analysis in early differential diagnosis of ovarian cancer is shown in Figure 1.

## 3. Method

At present, pharmaceutical companies not only focus on the molecular structure of drugs for drug design and *R*&*D* at the molecular level but also integrate the information related to drugs at a higher level, discover the mechanism of drug action, and improve the efficiency of drug *R*&*D* [11]. With the development of systems biology, drugs are no longer regarded as an isolated chemical molecule. They are related to many substances in the human body and exchange information, such as proteins, cells, and tissues. Drug therapy can be seen as a kind of disturbance to human physiological function at the system level [12]. Through this disturbance, human function changes towards a healthy state. To study drugs based on the viewpoint of systems biology, it is necessary to integrate multiple levels and multilevel information to characterize the characteristics of drugs, such as molecular level, cell level, organization level, individual level, and population level. This poses a great challenge to the current drug data mining methods, mainly reflected in the following aspects: data nonlinearity. Due to the complex pathogenesis, drug treatment is an extremely complex nonlinear process, which requires complex nonlinear methods to simulate the treatment mechanism of drugs and study different data structure types. Substances related to drug information often involve different data structures, and they are often stored in different databases [13]. Because different databases store data in different ways, it poses a great challenge for us to extract useful drug feature information. For example, the data description of biological databases often focuses on string sequence (protein sequence and gene sequence), text (gene ontology and functional site description), numerical value (composition and physical and chemical constants), graph (three-dimensional structure), etc. [14, 15]. Chemical database descriptions are often based on string (SMILES format), text (MOL file, SDF), numerical value (physical and chemical constants), graph (molecular structure), etc. In addition, there are some drug and protein enzyme classification and description methods, such as drug ATC classification system and EC classification system, which are characterized by text. These different data descriptions can provide rich characteristic information for drugs [16]. However, how to extract these features effectively is very difficult. At present, the frequently used numerical characterization is far from meeting the needs of drug information processing, so more effective methods are needed for extraction of this nonnumerical feature information and data fusion. For the above-mentioned drug-related information, they reflect the behavior of drugs from different aspects. Integrating this information together will help us understand the behavior of drugs from a systematic perspective [17]. However, in the face of such complex and huge data resources, how to integrate them in an effective way is an urgent problem to be solved [18]. The emergence and development of nuclear methods can solve the above problems to a certain extent. As introduced in the Introduction, the kernel method can effectively deal with nonlinear problems in data by constructing a suitable kernel function such as Gaussian kernel function and polynomial kernel function. Many theoretical and experimental studies show that the kernel method has excellent performance and flexibility in dealing with nonlinear data. In addition, by constructing different kernel functions, such as text kernel, string kernel, graph kernel, and tree kernel, the kernel method can effectively deal with various types of data, including numerical and nonnumerical, which greatly reflects the flexibility of the kernel method. More importantly, through the fusion of kernel functions, different types of data can be effectively integrated together, so that a multilevel model can be established at the system level to understand the mechanism of drug action. A support vector machine (SVM) is a standardized identification algorithm based on the principle of standardized risk reduction in representation science [19]. In the case of linear separation, SVM divides the height of the center by creating a hyperplane of the upper class. Suppose the dataset is {(*x*_*i*_, *y*_*i*_)}_*i*=1_^*N*^, where *x*_i_ is the ith sample vector and *y*_i_ is the category label of the ith sample. Then, the decision function of SVM can be expressed as

(1) $$\begin{array}{c} f\left(x_{i}\right)=Sgn\left(w^{t}x_{i}+b\right)\text{.} \end{array}$$

Here, *W* is the weight vector and *b* is the constant term. First, the conditions for proper assignment can be shown as

(2) $$\begin{array}{c} y_{i}\left[w^{t}x_{i}+b\right]\geq 1\text{.} \end{array}$$

SVM aims to find the weight vector *W* and the constant term *b* by minimizing ‖*w*‖^2^.The final decision function of SVM can be expressed as

(3) $$\begin{array}{c} f\left(x\right)=Sgn\left[\overset{N}{\underset{i=1}{\sum }}y_{i}\alpha_{i}K\left(x_{0},x_{i}\right)+b\right]\text{.} \end{array}$$

Here, *K*(*x*, *x*_*i*_) is a kernel function that determines the inner product between two samples in a given space and *α*i is a pair of variables. Different functions can be designed to meet different needs. We will then construct the kernel function of the line from the image of the SMILES chain to determine the molecular similarity. We can determine the kernel matrix by computing the inner product of their subrows. In other words, the string kernel can be defined by the inner product of the substring frequency. More precisely, assuming two strings S and *T*, whose substring frequencies are *φ*(*s*) and *φ*(*t*), respectively, the string core can be defined as

(4) $$\begin{array}{c} k\left(s,t\right)=＜\varphi \left(s\right)，\varphi \left(t\right)＞\text{.} \end{array}$$

Five datasets were extracted from the DSSTox database. They are DBPCANN data, Center data, EPAFHM data, CPDBAS data, and FDAMDD data. A summary of the five datasets used in this study is listed in Table 1.

In this study, C-SVM is used to create a classification model. In the SMILES string kernel-based C-SVM, two parameters need to be optimized: the control parameter C and the minimum line length P. Non-C controls keep class boundaries balanced and reduce class errors. If C is too low, we will not be able to include enough data. If C is too large, the model will fit in the training file. The control parameter C should be optimized by the selection method. The minimum wire length P is used to form the core wire. For example, if *p* = 2, all lines with *P* ≥ 2 are used to form the kernel matrix. We can also see that SVM based on SMILES string kernel seems to achieve relatively poor prediction accuracy on the EPAFHM dataset, as shown in Table 2.

The ROC curve is predicted by SVM based on SMILES string kernel on five datasets, as shown in Figure 2.

To further verify the predictability of our model, we split the entire dataset into 75% training packets and 25% independent validation packets based on row spacing. The prediction results for the five datasets on the independent validation package are listed in Table 3.

To further test the core performance of SMILES circuits, five datasets are classified using commonly used molecular determinants, such as molecular composition determinants, topological structural determinants, topochemical determinants, and electronic state determinants. A total of 223 molecular definitions will be calculated using our Cem package. Before creating the template, a series of descriptor selection steps will be performed with caret package in *R* language: remove those descriptors whose descriptor values are close to 0 or zero variance and subtract one of the two determinants with a correlation coefficient greater than 0.95; the significance of each determinant is assessed by the area under the ROC curve, excluding molecular determinants with a significance less than 1.5 [20, 21]. Finally, residual molecular determinants are used as distribution models. C-SVM with Gaussian kernel function is used to create the classification model. Both parameters (tuning parameter C and kernel parameter sigma) are optimized with network input. The optimal performance on the five datasets is as follows: for DBPCANN data, *C* = 100, sigma = 0.0141; for Center data, *c* = 1, sigma = 0.0187; for EPAFHM data, *c* = 1, sigma = 0.0174; for CPDBAS data, *c* = 10, sigma = 0.0198; and for FDAMDD data, *c* = 10, sigma = 0.015. The prediction results of the 5-fold interactive test on 5 datasets are listed in Table 4.

In this section, we aim to construct an informative string kernel function with the help of SMILES characterization of chemical molecules and use it in combination with the SVM algorithm to predict the toxicity of compounds. Like the UPAC chemical name of chemical molecules, its SMILES format can characterize the information of molecular structure, such as chemical element composition, valence bond information, and ring information. Therefore, it is feasible to construct chemical molecular similarity directly based on SMILES strings. Assuming that the model needs to be isolated, the k-NN algorithm selects K models that are similar to the model that needs to be isolated through the training process and then estimates the model K based on class voting or weight metrics. The Euclidean distance or other distance measure is usually chosen to measure consistency. The k-NN kernel algorithm is a continuation of the original k-NN algorithm. Its first plot shows the data through nonlinear mapping into a high-frequency field, followed by a k-NN model in this high-frequency field. Assume that the training data are as follows:

(5) $$\begin{array}{c} D=\left\{\left[x_{1},y_{1}\right],\ldots \ldots ,\left[x_{n},y_{n}\right]\right\}\text{.} \end{array}$$

We first map the training data to a feature space, as shown by

(6) $$\begin{array}{c} =\left\{\left[\phi \left(x_{1}\right),y_{1}\right],\ldots \ldots ,\left[\phi \left(x_{n}\right),y_{n}\right]\right\}\text{.} \end{array}$$

To get the k-NN algorithm, the key problem is how to calculate the Euclidean distance between two samples *ϕ*(*x*_*i*_)=*i* ∈ (1,2,…, *n*) and *ϕ*(*x*_*j*_) in the feature space.

The Euclidean distance between the training sample *ϕ*(*x*_*i*_) and the sample *ϕ*(*x*) to be classified can be expressed as

(7) $$\begin{array}{c} Dis=\sqrt{{\left\|\phi \left(x_{i}\right)-\phi \left(x\right)\right\|}^{2}}\\ =\sqrt{A-2B+C}\text{.} \end{array}$$

Here, *A* is *K*(*i*, *i*); *B* is the inner product between the training sample *ϕ*(*x*_*i*_) and the sample to be classified *ϕ*(*x*), which can be calculated by applying the kernel function to the training sample and the sample to be classified; and C is the inner product of the sample *ϕ*(*x*) to be classified, which can be calculated by mapping the kernel function to the test sample. The significance of each determinant was assessed by the area under the ROC curve, excluding molecular determinants with a significance less than 1.5. The remaining molecular determinants were used to create a classification model. For these three datasets, the remaining molecular identifiers are 47, 58, and 37, respectively. To test the predictability of the kernel's k-NN model, a comparison of Gaussian kernel-based SVMs was performed, and a five-fold interaction test was performed to evaluate the predictability of the two methods. All parameters were optimized by the lattice search strategy. The prediction results of the 5-fold interactive test of the two modeling methods are shown in Table 5.

With the first three datasets, we validate k-NN kernel performance on vectorized data. Next, we will give an example of k-NN on nonvectorized data. Primary advanced testing (PCA) is a process of eliminating design data from quality data. For p-dimensional X-matrix data, multiple orthogonal directions (loading matrix V) can be computed. In real problems, we need to use some components to determine most of the data variability. That is to say, we use the first *k* directions (i.e., VK) to try to reconstruct new data that maintain the original data structure. For the original PCA algorithm, we can calculate its covariance matrix, as shown by

(8) $$\begin{array}{c} C=\frac{1}{n}\overset{n}{\underset{i=1}{\sum }}x_{i}x_{i}^{t}=\frac{1}{n}x^{t}x\text{.} \end{array}$$

The principal component V can be calculated by solving the following eigenvalue problem:

(9) $$\begin{array}{c} \lambda v=Cv=\frac{1}{n}X^{t}Xv\text{.} \end{array}$$

Here, *λ*＞0 an d *v* ≠ 0; the feature direction corresponding to all nonzero eigenvalues can most support the same space as the original data matrix *X*, so the feature vector V can be re-expressed as

(10) $$\begin{array}{c} v=\overset{n}{\underset{i=1}{\sum }}\alpha_{i}x_{i}=X^{t}\alpha . \end{array}$$

Here, *α*=[*α*_1_,…*α*_*n*_]^*t*^; the eigenvalue problem can be re-expressed as

(11) $$\begin{array}{c} \lambda \alpha =\frac{1}{n}K\alpha . \end{array}$$

Here, *K* is a linear kernel function. In order to obtain the characteristics of a new sample *x*, we can simply map *φ*(x) to the first *k* directions VK, as shown by

(12) $$\begin{array}{c} v_{k}•\phi \left(x\right)=\overset{n}{\underset{i=1}{\sum }}\alpha_{i}^{k}＜\phi \left(x_{i}\right),\phi \left(x\right)＞=\overset{n}{\underset{i=1}{\sum }}\alpha_{i}^{k}k\left(x_{i},x\right)=k_{test}•\alpha \text{,} \end{array}$$

where

(13) $$\begin{array}{c} k_{test}=M•\phi \left(x\right)\text{.} \end{array}$$

For nonlinear classification, the basic SVM first maps the data in the space to the high points of the kernel function by defining a kernel function and then completes the LSVM algorithm here. However, if the variables in the kernel space are redundant or noisy, it may affect the accuracy of the model assumptions, so that unnecessary information must be removed before running the LSVM algorithm. To deal with this situation, we coupled KPCA and LSVM algorithms to generate a two-step nonlinear algorithm (KPCA + LSVM). KPCA + LSVM algorithm steps are shown in Figure 3.

In this section, a two-step nonlinear classification algorithm KPCA + LSVM is developed to model the structure-function relationship. For the KPCA + LSVM algorithm, KPCA can effectively capture the underlying data structure in the kernel function space by removing noninformative components. LSVM can build a powerful classifier in KPCA transformed feature space by maximizing the boundary hyperplane. Compared with the LSVM algorithm and the other two nonlinear methods, KPCA + LSVM can effectively improve the prediction performance of the model by processing the redundant information in the kernel feature space. When all principal component scores are used to construct the kernel matrix, the algorithm is consistent with the current nonlinear SVM algorithm. The application of KPCA + LSVM algorithm on three activity relationship data fully proves that the two-step algorithm is a promising modeling method in drug research [22].

## 4. Experiment and Analysis

There is no effective treatment for hospital-acquired ovarian cancer. We screen the potential therapeutic drug sanguinarine for cisplatin resistance of ovarian cancer by bioinformatics methods. In this section, the MTT method is used to investigate the effect of sanguinarine on cisplatin against COC1/DDP of ovarian cancer, and to provide experimental basis for further study of sanguinarine in the prevention of ovarian cancer in medicine [23, 24]. In the process of drug data mining, learning algorithms often face the problem of selecting compact feature subsets. In practice, there are many reasons for feature selection: a large number of features often introduce unnecessary noise into the model, thus affecting the prediction accuracy of the model. When the model contains many features, it is difficult to determine which features or feature combinations contribute to the prediction of the model, which brings great difficulties to explain the model. Biological and medical research requires us to identify the highest ranked features, which can provide guidance for drug research. In terms of computational efficiency, we need more time to establish prediction models with many characteristics. The existence of a large number of features may cause the model to be unstable or even not work properly [25]. If the number of features significantly exceeds the number of samples, or there are multiple linear connections between attributes, data overfitting often occurs, which will seriously affect the prediction performance of the model, resulting in invalid prediction models. At present, integrated learning algorithms based on decision tree, such as bagging, boosting, and random forest, have been widely used in the field of chemistry and pharmaceutical research. These methods improve the prediction accuracy of the model by combining multiple decision tree models. They overcome the shortcomings of a single decision tree model (low accuracy and instability) but maintain the advantages of the decision tree model. In addition, the decision tree-based ensemble learning algorithm can easily sort features. However, whether these decision tree-based ensemble learning algorithms still suffer from feature selection is still worth studying. Previous studies have shown that when the data include no information or noise features, the prediction accuracy of a single decision tree model will also be affected. In this section, we study the feature selection problem based on the decision tree ensemble learning algorithm. We propose an automatic consequent elimination strategy to select a compact subset of features step by step. Six SAR datasets related to drug ADMET were used to confirm the rationality of our method. We construct a generalized variable selection framework based on the backward elimination strategy (BES). The flow chart of variable selection based on the decision tree integration algorithm is shown in Figure 4.

The BES basically consists of the following three sequential steps. In the first step, a hypothesis model is developed using a decision tree-based ensemble algorithm, and the saliency and loss functions of the corresponding variables are calculated. The loss function is defined as

(14) $$\begin{array}{c} {Fittness}_{i}=\frac{1}{10}\overset{10}{\underset{k=1}{\sum }}error_{k}+\lambda \left|p_{i}\right|\text{.} \end{array}$$

In the second step, an exponential decay function is used to eliminate variables with small importance. In the ith iteration, the proportion of the reserved variables can be calculated by the exponential decay function, as shown by

(15) $$\begin{array}{c} r_{i}=a*\exp\left(-K*i\right)\text{.} \end{array}$$

Here, *a* and K are two constants of the exponential decomposition function, which can be determined by the following two conditions. *r*_*i*_ is 1 if all variables are included in the model. If only 5% of the variables are stored in iteration B, *r*_*B*_ = 5% can be calculated based on the two conditions a and K, as in the following equations:

(16) $$\begin{array}{c} a={\left(r_{B}\right)}^{1/\left(B-1\right)}\text{,} \end{array}$$

(17) $$\begin{array}{c} k=-1n\left(\frac{\left(r_{B}\right)}{B-1}\right)\text{.} \end{array}$$

In the third step, after B iterations, we can obtain B variable subsets and B loss functions. We can determine a learning curve according to these B loss functions. Typically, the learning curve will be too lower first, reach the lowest point, and then rise again. We can choose different subsets with the smallest loss rate as the final selected subset difference. In general, a selection algorithm usually requires three main factors: the design model, the research philosophy, and the functional goals, to lead the research. In this study, the integrated method based on decision trees is used to build the mathematical model. The search algorithm uses the strategy of gradual elimination of subsequent items. In addition, the use of exponential decay function effectively overcomes the low efficiency of the latter elimination strategy [26]. The objective function that guides the search plays a key role in variable selection. In this study, it consists of two items: the average value of the error rate of the interactive test and the penalty term. We first evaluate and compare the prediction performance of different decision tree integration methods on all descriptors. Five interaction tests were used to evaluate the predictive performance of various ensemble methods. As for the wheelchair method, we use the Gini net criterion to partition the decision tree. For the bundled and RF methods, we create a predictive model using the sum of 500 decision trees. In addition, mtry is an important parameter that affects RF prediction. According to Breiman, the RF model achieves better performance by choosing mtry as the square root of all functions. In this study, we chose the values proposed by Breiman to create the model. For support, the best tree set is determined by a 5-fold interaction test. In order to make our prediction results more reliable, we randomly repeated the 5-fold interaction test for ten times, and the average prediction for ten times was used as the comparison standard of different integration methods. The prediction results of different decision tree integration methods on all descriptors are listed in Table 6.

The prediction performance of the integrated method based on the BES with variable selection is significantly better than that of the integrated method without variable selection. The same is true for each dataset. This implies that variable selection can indeed improve the prediction performance of the decision tree ensemble method. The boosting model without BES is worse than the bagging model with the BES, which shows that the decision tree integration method also suffers from the disaster of dimensionality to a certain extent. For each data, the prediction results are consistent with the average prediction accuracy. Although various decision tree integration methods have variable selection mechanisms, the application of additional variable selection procedures is also very important in decision tree integration methods. Among the three integration methods, boosting achieves the BES prediction performance again [27, 28]. There is no significant difference in performance between bagging with the BES and RF. This may be because the descriptors selected by the BES are not related. The RF model reduces the correlation between decision trees by selecting some variables, which improves the prediction performance of bagging. Therefore, when the descriptors selected by the BES are uncorrelated, the RF model does not show greater advantages. In a word, the prediction performance of the three decision tree integration methods is greatly improved by using the BES to select variables. The prediction results of different decision tree integration algorithms on the two feature sets are shown in Table 7.

It can be seen that compared with the RF model, the fisaRF model has significantly improved the prediction performance. It achieved 85.77% prediction accuracy, 90.45% sensitivity, 73.47% specificity, and 66.08% Matthews correlation coefficient [29]. All these statistics are better than the RF corresponding statistics. For one-shot data, fisaRF also accomplishes better estimation performance than RF, implying that fisaRF improves RF prediction rather than being different by the nature of data sharing. A good distribution model must not only have good isolation but also be reliable in advance. A high prediction confidence indicates that the compound is more likely to be classified.

DBPCANN data with different numbers of identifiers were used to assess the predictability of fisaRF. We first counted 1,458 distinct molecular identifiers, including 1,020 fingerprints without complete information and 438 nonzero identifiers. Finally, 153 descriptors were extracted from these feature sets. In this way, we used 1548, 438, and 153 descriptors to characterize DBPCANN data. Here, we use the 00B error estimation method with RF itself to evaluate the prediction accuracy of the model. In order to obtain more reliable predictions, we repeatedly established 20 models to obtain the mean value of these prediction statistics. Obviously, fisaRF achieves better prediction performance. The increased uniqueness is even more amazing. An important conclusion is that fisaRF appears to be insensitive to changes in the number of determinants. There was no statistical difference between the two methods. The fisaRF and RF classification results on DBPCANN data are shown in Table 8.

For an in-depth comparison, we also calculated the AUC values of fisaRF and RF on different sets of functions. The sensitivity and specificity of fisaRF and AUC were significantly higher than those of RF. For three different sets of functions, fisaRF achieved AUCs of 98.19%, 98.08%, and 98.05%, respectively. MCTree mainly embodies the idea of uniform selection of variables. Since the sampled similarity matrix on MCTree consists of a series of models of decision tree, the variability of MCTree can be determined by summing the variables of all models of decision tree. The calculation formula is shown as

(18) $$\begin{array}{c} J\left(i\right)=\frac{1}{ntree}\overset{ntree}{\underset{b=1}{\sum }}J_{M_{b}}. \end{array}$$

Here, ntree is the number of decision tree models to be established. Mb is the b-th decision tree. Mb(i) is the significance of variable *i* of decision tree *b*. Determining the significance of a difference in tree structure depends on the reduction in purity of all nonterminal nodes using that difference. In this way, the value of each mean difference gets the difference in MCTree [30]. The blending option ensures that the switching options of the MCTree model actually affect the contribution to the distribution, not the environment. Therefore, the switches selected by MCTree are stable and reliable. Suppose the *X*-matrix data model includes *n* and P difference vectors, and the *y* difference response is an n-dimensional vector. For binary classification problems, the element of Y is +1 or -1. Fisher discriminant function can be expressed as

(19) $$\begin{array}{c} y=\text{sgn}\left(w^{t}x+b\right)\text{.} \end{array}$$

A newly developed KFDA method was used to classify rapid and nondestructive data on blood glucose. In KFDA, the number of tuning trees is set to nti = 400. The values of *R* and tuning parameter *f* can be found in the search grid (*R* = 0.5 and *λ* = 11) holding and snip. For each tree determination, 50% of the material was used to create the design template and the other 50% was used for pruning. The prediction kernel matrix KT collects the similarity information between training samples and test samples. The KFDA method obtained 94.83% prediction accuracy, 87.5% sensitivity, and 100% specificity, respectively.

The drug resistance of ovarian cancer cells is a major difficulty in the treatment of ovarian cancer. There is no effective treatment for drug-resistant ovarian cancer in clinic. We screened the potential therapeutic drug sanguinarine for cisplatin resistance of ovarian cancer by bioinformatics methods. In this part, the effect of sanguinarine on the cisplatin-resistant ovarian cancer cell line coc1/ddp will be preliminarily verified by the MTT method, so as to provide an experimental basis for the in-depth study of sanguinarine in cisplatin-resistant ovarian cancer. Sanguinarine can inhibit the growth of cisplatin-resistant ovarian cancer coc1/ddp cell line, and the inhibition rate increases with the increase of time and drug concentration. The results are shown in Table 9.

Ovarian cancer is a common malignant tumor with the highest mortality rate in gynecology. Its early diagnosis is difficult. Most patients with ovarian cancer are found to be in the advanced stage, and surgery alone cannot achieve good therapeutic effect. Therefore, chemotherapy is a necessary and important measure for the treatment of ovarian cancer. The chemotherapy cycle for ovarian cancer is longer than that for other women's cancers, and early chemotherapy for ovarian cancer makes the widely used ovarian cancer cells more likely to develop drug resistance. How to reverse the resistance of ovarian cancer to chemotherapy has become a major topic of ovarian cancer treatment. In bioinformatics research, we found that sanguinarine may be a potential drug for the treatment of drug-resistant ovarian cancer, and sanguinarine is low cost and has a wide range of sources and few toxic and side effects. Therefore, we selected sanguinarine as a research object in the treatment of drug-resistant ovarian cancer [31, 32].

## 5. Conclusion

Ovarian cancer is one of the most common cancers in pregnant women with high mortality. Most ovarian cancer patients are diagnosed at an advanced stage because the initial symptoms of the disease are unknown. Furthermore, ovarian cancer has a very poor prognosis due to its high recurrence rate and resistance to chemotherapy. Therefore, ovarian cancer has been paid more and more attention in the research of gynecological tumors, especially ovarian serous cystadenocarcinoma in recent years. At present, this field focuses on the study of the mechanism of ovarian cancer occurrence, development, and metastasis, in order to provide new ideas and new methods for the early diagnosis and clinical treatment of ovarian cancer. lncRNA is an endogenous noncoding RNA with a length more than 200 nt. It has a high degree of tissue and physical and spatial specificity and can regulate gene expression levels at various stages (epigenetic regulation, transcriptional regulation, posttranscriptional regulation, etc.). In recent years, some lncRNAs have been found to be related to the occurrence, development, and metastasis of ovarian cancer, but their molecular mechanisms are still unclear. In addition, there are a large number of ovarian cancer disorders lncRNA function that has not been found. With the accumulation of transcriptome data of ovarian cancer and the implementation of cancer gene mapping (TCGA) program in recent years, we have been able to study the function and molecular mechanism of ovarian cancer-related lncRNA through systems biology and bioinformatics methods. This paper mainly solves some problems in the field of lncRNA recognition and function research by developing new bioinformatics tools and databases, enriches the methods of lncRNA research, and finally constructs the lncRNA regulatory network through the analysis of high-throughput transcriptome sequencing data of ovarian cancer, so as to analyze the potential function and mechanism of lncRNA in ovarian cancer.

## Figures and Tables

**Figure 1:** Role of bioinformatics analysis in early differential diagnosis of ovarian cancer.

**Figure 2:** ROC curve predicted on five datasets by SVM based on SMILES string kernel.

**Figure 3:** KPCA + LSVM two-step algorithm flow chart.

**Figure 4:** Flow chart of variable selection based on the integrated algorithm of decision tree.

**Table 1:** Summary of five datasets used in this study.

Data name	Nature of measurement	Number of molecules	Category 1	Category 2
DBPCANN	Evaluation of carcinogenicity of disinfectant	182	77	96
Center	Androgen receptor binding	222	137	92
EPAFHM	Acute toxicity of black-headed minnow	589	301	287
CPDBAS	Carcinogenic intensity	665	319	346
FDAMDD	Maximum recommended daily human dose	803	361	452

**Table 2:** Prediction results of the 5-fold interactive test of SVM based on SMILES string kernel on five datasets.

Dataset	TP	FN	TN	FP	SE	SP	ACC	MCC	AUC
DBPCANN	78	3	54	12	97.77	88.67	86.21	81.47	89.39
Center	124	20	88	19	84.74	88.49	90.22	70.08	97.01
EPAFHM	214	67	187	112	75.72	64.54	70.02	42.02	84.87
CPDBAS	264	92	276	65	69.36	82.68	72.34	54.05	87.04
FDAMDD	278	84	325	91	79.17	79.67	77.98	66.01	89.37

**Table 3:** Prediction results of SVM based on SMILES string kernel on the independent verification set.

Dataset	TP	FN	TN	FP	SE	SP	ACC	MCC	AUC
DBPCANN	21	4	17	1	91.78	89.04	89.71	82.01	89.71
Center	38	6	13	5	87.12	72.47	87.01	34.27	88.71
EPAFHM	43	19	42	24	76.37	63.24	70.01	40.24	74.14
CPDBAS	57	21	68	18	72.01	80.99	72.41	57.14	82.27
FDAMDD	84	37	73	21	78.04	76.27	78.01	57.34	87.01

**Table 4:** Prediction results based on the 5-fold interaction test and common molecular descriptors.

Dataset	TP	FN	TN	FP	SE	SP	ACC	MCC
DBPCANN	87	8	64	7	97.14	87.97	91.31	86.29
Center	148	14	67	104	88.17	74.77	84.87	66.39
EPAFHM	207	71	169	102	73.24	65.37	70.29	40.41
CPDBAS	227	78	247	79	73.87	72.24	76.24	50.27
FDAMDD	249	91	347	67	73.87	83.17	77.24	58.14

**Table 5:** Prediction results of the new interaction test of two modeling methods.

Dataset	TP	FN	TN	FP	SE	SP	ACC	MCC	AUC
HIA	114	16	40	25	87.70	61.54	78.97	51.29	84.43
	110	20	44	21	84.62	67.69	78.97	52.52	83.78

P-gP	98	17	67	18	85.22	78.82	82.50	64.14	86.99
	98	17	62	23	85.22	72.94	80.00	58.81	85.94

TdP	52	33	239	36	61.18	86.91	80.83	47.52	83.31
	43	42	252	23	50.59	91.64	81.94	46.43	81.85

**Table 6:** Prediction results of different decision tree integration methods on all features.

Dataset	CART	Bagging	RF	Boosting
HIA	72.87 (2.81)	78.37 (1.79)	79.64 (1.09)	80.57 (1.77)
P-gP	68.79 (2.87)	79.15 (2.77)	80.19 (1.71)	81.01 (1.57)
TdP	81.01 (1.21)	83.17 (0.81)	83.63 (0.37)	84.40 (0.34)
MDRR	77.33 (1.88)	82.44 (0.73)	83.14 (0.57)	83.47 (0.37)
BBB	72.07 (2.21)	76.01 (1.01)	76.03 (1.19)	78.72 (0.67)
Factor Xa	92.21 (0.91)	94.72 (1.12)	93.44 (0.55)	95.37 (0.49)
Average	77.03	82.34	82.64	83.77

**Table 7:** Prediction results of the decision tree integration method on different feature sets.

Dataset	All descriptors	Select descriptor	All descriptors	Select descriptor	All descriptors	Select descriptor
HIA	78.17	82.34	79.74	82.15	80.78	84.31
P-gP	79.23	81.74	80.15	82.74	80.71	81.89
TdP	83.14	85.24	83.13	84.52	84.14	87.65
MDRR	81.99	83.41	83.05	83.17	83.84	85.49
BBB	75.97	81.05	78.13	78.99	79.68	80.17
Factor Xa	93.17	95.40	92.19	95.54	94.34	96.17
Average	82.97	83.77	81.78	84.88	81.95	85.12

**Table 8:** Prediction results of fisaRF and RF on DBPCANN data.

Number of descriptors	Prediction accuracy		Sensitivity		Specificity		MCC value		AUC	
	RF	fisaRF	RF	fisaRF	RF	fisaRF	RF	fisaRF	RF	fisaRF
153	90.41	92.21	87.18	84.17	92.42	97.17	77.81	84.21	96.87	97.11
438	88.09	91.08	85.63	89.02	87.67	96.71	79.32	84.27	97.03	97.78
1458	88.12	92.27	87.51	87.17	90.27	97.37	78.88	85.10	95.29	98.15

**Table 9:** Inhibitory rates of sanguinarine and cisplatin on coc1/ddp cell lines.

Inhibition rate (%)			
Concentration (umol/l)	24 h	48 h	72 h
0	0.91 ± 0.13	1.39 ± 0.17	1.77 ± 0.26
1	5.30 ± 2.03^∗^	11 68 ± 0.92^∗^	17.48 ± 1.57^∗^
2	23.31 ± 2.39^∗^	29.93 ± 1.54^∗^	34.00 ± 1.59^∗^
3	30.72 ± 1.41^∗^	41.02 ± 1.70^∗^	56.65 ± 3.08^∗^
4	64.44 ± 4.40^∗^	62.35 ± 3.21^∗^	70.73 ± 1.71^∗^
5	83.55 ± 4.52^∗^	87.44 ± 2.15^∗^	95.37 ± 2.13^∗^

## Data Availability

No data were used to support this study.

## References

[1] Medhat B., Shawish A. (2020). ACCepted [early ACCess articles in ieeexplore] flr: a revolutionary alignment-free similarity analysis methodology for dna-sequences. *IEEE/ACM Transactions on Computational Biology and Bioinformatics*.

[2] Covington L. B., Patterson F., Hale L. E. (2021). The contributory role of the family context in early childhood sleep health: a systematic review. *Sleep Health*.

[3] Jiang W., Zhang C., Kang Y., Li G., Feng Y., Ma H. (2021). The roles and mechanisms of the circular rna circ_104640 in early-stage lung adenocarcinoma: a potential diagnostic and therapeutic target. *Annals of Translational Medicine*.

[4] Li Y., Tan Y. (2021). Bioinformatics analysis of cerna network related to polycystic ovarian syndrome. *Computational and Mathematical Methods in Medicine*.

[5] Wang Y., Yang Y., Na S., Liu T., You Y. (2020). Melatonin attenuates early brain injury via regulating mir-181a/tnf-*α*/nf-*κ*b signaling pathway following subarachnoid hemorrhage in rat. *Acta Medica Mediterranea*.

[6] Wu K. Z., Zhang C. D., Zhang C., Dai D. Q. (2020). A novel three-mirna signature identified using bioinformatics predicts survival in esophageal carcinoma. *BioMed Research International*.

[7] Cheng S., Song Q., Yu T. (2020). Characterization and expression analysis of four members genes of flavanone 3-hydroxylase families from chamaemelum nobile. *Notulae Botanicae Horti Agrobotanici Cluj-Napoca*.

[8] Liang Y., Zhu H., Chen J., Lin W., Li B., Guo Y. (2020). Construction of relapse-related lncRNA-mediated cerna networks in hodgkin lymphoma. *Archives of Medical Science*.

[9] Gisonno R. A., Masson T., Ramella N. A., Barrera E. E., Romanowski V. ., Tricerri M. A. (2022). Evolutionary and structural constraints influencing apolipoprotein a-i amyloid behavior. *Proteins: Structure, Function, and Bioinformatics*.

[10] Deng H., Huang Y., Wang L., Chen M. (2020). High expression of ubb, rac1, and itgb1 predicts worse prognosis among nonsmoking patients with lung adenocarcinoma through bioinformatics analysis. *BioMed Research International*.

[11] Fan X., Hao Z., Li Z., Wang X., Wang J. (2020). Inhibition of mir-17∼92 cluster ameliorates high glucose-induced podocyte damage. *Mediators of Inflammation*.

[12] Sung S. F., Lee P. J., Hsieh C. Y., Zheng W. L. (2020). Medication use and the risk of newly diagnosed diabetes in patients with epilepsy: a data mining application on a healthcare database. *Journal of Organizational and End User Computing*.

[13] Khalaf O. I., Abdulsahib G. M. (2021). Optimized dynamic storage of data (ODSD) in IoT based on blockchain for wireless sensor networks. *Peer-to-Peer Netw. Appl.*.

[14] Huang R., Zhang S., Zhang W., Yang X. (2021). Progress of zinc oxide-based nanocomposites in the textile industry. *IET Collaborative Intelligent Manufacturing*.

[15] Cao M., Zhang P. B., Wu P. F. (2021). Duox2 as a potential prognostic marker which promotes cell motility and proliferation in pancreatic cancer. *BioMed Research International*.

[16] Li M., Zhu Y., Tang L. (2021). Protective effects and molecular mechanisms of achyranthes bidentata polypeptide k on schwann cells. *Annals of Translational Medicine*.

[17] Li L, Diao Y., Liu X. (2014). Ce-Mn mixed oxides supported on glass-fiber for low-temperature selective catalytic reduction of NO with NH3. *Journal of Rare Earths*.

[18] Khalaf O. I., Abdulsahib G. M. (2020). Energy efficient routing and reliable data transmission protocol in WSN. *International Journal of Advances in Soft Computing and Its Applications*.

[19] Sengan S., Khalaf O. I., Rao G. R. K., Sharma D. K., Amarendra K., Hamad A. A. (2022). Security-aware routing on wireless communication for E-health records monitoring using machine learning. *International Journal of Reliable and Quality E-Healthcare*.

[20] Mao L., Ling X., Chen J. (2021). Cyclin h regulates lung cancer progression as a carcinoma inducer. *Computational and Mathematical Methods in Medicine*.

[21] Chen Y., Li J., Ouyang S., Luo L. (2020). Differentially expressed genes analysis on the role of wnt5a in lentoid body induction from human embryonic stem cells. *Zhonghua Shiyan Yanke Zazhi/Chinese Journal of Experimental Ophthalmology*.

[22] Gu J., Wang W., Yin R., Truong C. V., Ganthia B. P., Ganthia B. P. (2021). Complex circuit simulation and nonlinear characteristics analysis of GaN power switching device. *Nonlinear Engineering*.

[23] Jahangirimoez M., Medlej A., Tavallaie M., Mohammad Soltani B. (2020). Hsa-mir-587 regulates tgf*β*/smad signaling and promotes cell cycle progression. *Cell Journal*.

[24] Zhang Z., Wang J., Mao J., Li F., Chen W., Wang W. (2020). Determining the clinical value and critical pathway of gtpbp4 in lung adenocarcinoma using a bioinformatics strategy: a study based on datasets from the cancer genome atlas. *BioMed Research International*.

[25] Yuvaraj N., Srihari K., Dhiman G. (2021). Nature-inspired-based approach for automated cyberbullying classification on multimedia social networking. *Mathematical Problems in Engineering*.

[26] Gubkina M. F., Yukhimenko N. V., Petrakova I. Y., Khokhlova Y. Y., Sterlikova S. S. (2020). The role of social factors in the development of chronic primary tuberculosis in early childhood. *Rossiyskiy Vestnik Perinatologii i Pediatrii (Russian Bulletin of Perinatology and Pediatrics)*.

[27] Kumalasari D., Fourianalistyawati E. (2020). The role of mindful parenting to the parenting stress in mothers with children at early age. *Jurnal Psikologi*.

[28] Ismagilov A. K., Khuzina D. R., Vanesyan A. S., Zaysteva V. V. (2021). The role of biomarkers in the early diagnostics of breast cancer. *Tumors of Female Reproductive System*.

[29] Pradeep Raj M. S., Manimegalai P., Ajay P., Amose J. (2021). Lipid data acquisition for devices treatment of coronary diseases health stuff on the internet of medical things. *Journal of Physics: Conference Series*.

[30] Hu X. L., Su Q., Meng d. L., Ren Y. S., Su Z. Q. (2021). Circular rna expression alteration and bioinformatics analysis in patients with acute cerebral infarction injury. *Bioengineered*.

[31] Lim C. K., Kim D. Y., Cho A., Choi J. Y., Park J. Y., Kim Y. M. (2021). Role of minimally invasive surgery in early ovarian cancer. *Gland Surgery*.

[32] Essmat A. (2021). Role of ovarian fertility sparing surgery (fss) in cases of early stage 1 ovarian cancer in patients in reproductive age group. *Open Journal of Obstetrics and Gynecology*.

